RETRACTED

# Preliminary Study on the Therapeutic Effect of Doxorubicin-Loaded Targeting Nanoparticles on Glioma

**DOI:** 10.1155/2022/6405400

**Published:** 2022-03-28

**Authors:** Weitu Lan, Hongguang Zhang, Bo Yang

**Affiliations:** ^1^Department of Neurosurgery, Cangzhou People's Hospital, Cangzhou, 061000 Hebei, China; ^2^Department of Neurosurgery, Gaotang People's Hospital, Liaocheng, 252800 Shandong, China; ^3^Department of Neurosurgery, Zibo Central Hospital, Zibo, 255000 Shandong, China

## Abstract

Doxorubicin (DOX) is an anthracycline anticancer drug, which is often associated with drug resistance and cytotoxicity. More unfortunately, the biological barrier in the human environment can weaken the efficacy of DOX, such as the blood-brain barrier (BBB). This work attempts to make efforts to solve this problem. We used polyethylene glycol distearoylphosphatidylethanolamine (PEG-DSPE) as a nanocarrier and DOX as a model drug to construct a composite nanodrug (TF-PEG-DSPE/DOX NPs) by coupling transferrin (TF). The results of glioma experiments show that the nanodrug can effectively penetrate BBB to achieve an antitumor effect.

## 1. Introduction

The rapid development of medical technology provides effective solutions for many clinical diseases. However, a radical cure for cancer has not been achieved in the current medical community. As a kind of malignant tumor that originated from the brain neuroectoderm, glioma has strong aggressiveness and high mobility. The five-year survival rate of patients is less than 10%, and the difficulty of treatment is self-evident [1–4].

At present, surgical resection is the first choice for the treatment of glioma at home and abroad, supplemented by radiotherapy and chemotherapy [5–8]. With the development of medical imaging technology (such as magnetic resonance imaging and stereotactic technology), the accuracy of surgical resection has been greatly improved, which provides the basis for the cure of glioma [9–12]. However, due to the infiltration and growth characteristics of glioma, even experienced surgeons cannot completely remove the lesions [13–16]. Radiotherapy is an effective means to improve the survival rate of cancer patients, which has been agreed upon by the medical community. However, it has been reported that the sensitivity of radiotherapy is different among individuals, which leads to the lack of guarantee of treatment effectiveness. In addition, studies have found that the clinical application of radiation is often accompanied by strong side effects (such as hair loss, skin allergy, and decreased immune function) [17]. Therefore, this work chose chemotherapy as the research direction, trying to find a kind of targeted drug with strong efficacy and lower side effects.

RETRACTED

DOX is a common antibiotic tumor drug, and its structure is shown in Figure 1. Clinical studies have shown that DOX has a significant toxic effect on breast cancer, lymphatic cancer, ovarian cancer, thyroid cancer, glioma, and other tumor cells [18–22]. At the same time, DOX can promote the formation of superoxide radicals and destroy the membrane structure of cancer cells. However, the existence of BBB on the surface of the body's brain tissue has greatly affected the DOX drugs [23–25]. Therefore, the development of DOX-targeted drugs is the primary problem.

Recently, some researchers have been inspired by the specific binding process between transferrin (TF) and its receptor. Overexpression of TF receptors in glioma cells greatly increases the ability of tumor drugs carrying TF to penetrate BBB [26–28]. Therefore, the development of effective antiglioma drugs containing TF is increasing. Among them, the research data of drug modification based on nanotechnology are numerous. Due to its unique size and excellent drug binding ability, the nanodrug delivery system provides a new opportunity for the efficient treatment of malignant glioma. Polyethylene glycol distearoylphosphatidylethanolamine (PEG-DSPE) is a derivative of polyethylene glycol (PEG), which contains both the hydrophilic and hydrophobic segments. Therefore, PEG-DSPE is very common as a nanodrug carrier [29, 30].

In this paper, DOX was used as a model drug to couple PEG-DSPE with TF, and novel doxorubicin-loaded nanoparticles (TF-PEG-DSPE/DOX NPs) were prepared. In addition, in order to investigate the antitumor effect of the nanoparticles, the *in vitro* and *in vivo* experiments of TF-PEG-DSPE/DOX NPs were carried out orderly (Figure 2).

## 2. Materials and Methods

### 2.1. Materials and Instruments

Polyethylene glycol phospholipid (PEG-DSPE, C_44_H_87_N_2_O_10_P) was purchased from Shenzhen Meiluo Technology Co., Ltd. (Guangdong, China). Doxorubicin (DOX, C_27_H_29_NO_11_) was purchased from Hubei Yongkuo Technology Co., Ltd. (Hubei, China). Dimethyl sulfoxide (DMSO, C_2_H_6_OS) was purchased from Shanxi Jinyang Pharmaceutical Excipients Co., Ltd. (Shanxi, China). Triethylamine (TEA, C_6_H_15_N) was purchased from Jinan Yeqing Biotechnology Co., Ltd. (Shandong, China). Transferrin (TF) was purchased from Shanghai Qiyuan Biotechnology Co., Ltd. (Shanghai, China). Brain endothelioma adherent cell line bEnd.3 and glioma cell line U87 were purchased from Shanghai Binsui Biotechnology Co., Ltd. (Shanghai, China). Thiazolyl blue (MTT, C_18_H_16_BrN_5_S) was purchased from Wuhan Kanos Technology Co., Ltd. (Hubei, China). Phosphate-buffered saline (PBS) was purchased from Shanghai Jizhi Biochemical Technology Co., Ltd. (Shanghai, China). Chloral hydrate (TCA, C_2_H_3_Cl_3_O_2_) was purchased from Shanghai Xinyu Biotechnology Co., Ltd. (Shanghai, China).

RETRACTED

The MR-96A microplate reader was purchased from Shenzhen Mindray Bio-Medical Electronics Co., Ltd. (Guangdong, China).

### 2.2. Preparation of TF-PEG-DSPE/DOX NPs

Weigh 1.0 g of PEG-DSPE and 250 mg of DOX and dissolve in 10.0 mL of DMSO solution. Add 0.10 mL of TEA solvent dropwise to the reaction system, then place at a 40°C water bath constant temperature shaker and wait for the reaction for one day to prepare a PEG-DSPE/DOX NP solution. Finally, TF was used to specifically bind the DSPE group of PEG-DSPE/DOX NPs by the TF thiolation method to obtain TF-PEG-DSPE/DOX NPs.

### 2.3. *In Vitro* Experiments

#### 2.3.1. Permeability of BBB Modulus

The performance of single DOX drugs, PEG-DSPE/DOX NPs, and TF-PEG-DSPE/DOX NPs in penetrating the blood-brain barrier was compared. Briefly, the logarithmic growth phase mouse brain endothelioma adherent cell line bEnd.3 was inoculated into the upper chamber of a 24-well plate Transwell with a concentration of 5.0 × 10^4^ cells/well and placed in the lower chamber containing 10% fetus. A fresh medium of bovine serum is cultivated. Closely observe the compactness of the cell monolayer. When the transmembrane resistance value of the monolayer cells is greater than 200 *Ω*/cm^2^, change the medium to a cell culture medium without fetal calf serum, and DOX, PEG-DSPE/DOX NPs, and TF-PEG-DSPE/DOX NPs were added to the upper chamber; 200 *μ*L of culture medium was removed every 6.0 h, and the same amount of fresh culture medium was replaced in the lower chamber. Use a microplate reader to detect the fluorescence intensity at 630 nm.

#### 2.3.2. Inhibitory Effect of Composite Nanodrugs on U87 Cells

The MTT method was used to evaluate the inhibitory effect of TF-PEG-DSPE/DOX NPs on the glioma cell line U87. Briefly, the diluted U87 cell suspension was seeded in a 98-well plate at a concentration of 1.0 × 10^4^ cells/well. After one day of culture, add 150 *μ*L of DOX, PEG-DSPE/DOX NP, and TF-PEG-DSPE/DOX NP solutions (5.0, 15, 25, 35, and 45 *μ*M). After the cells are cocultured with the drug for one day, add 25 *μ*L of MTT solution to the 96-well plate and incubate for 4.0 h. After removing the supernatant, add DMSO solution dropwise to the culture plate to stop the entire reaction system. Record the absorbance of the reaction products of each experimental group at 490 nm to obtain the inhibitory rate of the drug on U87 cells.

#### 2.3.3. *In Vitro* Drug Release

Use the dialysis method to explore the cumulative release of TF-PEG-DSPE/DOX NPs *in vitro*. Briefly, adjust the pH of the PBS = 7.4, and dissolve 10.0 mg of TF-PEG-DSPE/DOX NPs in the PBS. Place the dialysis bag in an incubator at a constant temperature of 37°C for continuous shaking, and collect at preset time points (0.5, 1.0, 2.0, 4.0, 6.0, 12, 24, and 48 h) 2.0 mL of dialysis external fluid, and use PBS to refill in time. The sample was filtered, and the drug release was determined by high-performance liquid chromatography.

RETRACTED

### 2.4. *In Vivo* Experiment

#### 2.4.1. Construction of the Glioma Model

In order to evaluate the targeted antitumor effect of TF-PEG-DSPE/DOX NPs, 84 BALB/c nude mice aged 6–8 weeks were selected as experimental subjects in this study. All mice were fasted and deprived of water within 12 h before the start of the operation and anesthetized by intraperitoneal injection of TCA (2.5 mL/kg). Fix the mouse on the stereotaxic device, and drill a 2.0 mm diameter hole on the midline of the forehead after skin preparation. Keep the microsyringe with a 5.0 mm needle, and then slowly inject 2.0 *μ*L of U87 cells in the logarithmic growth phase (concentration of 1.5 × 10^6^ cells/*μ*L) into the mouse brain. After 10 min of observation, slowly take out the microsyringe. The incision was sutured after washing and disinfection, and 1.5 × 10^5^ U penicillin was injected daily for preinfection within 7 d after surgery.

#### 2.4.2. Treatment Plan

After the glioma model was successfully induced, they were randomly divided into the DOX group, PEG-DSPE/DOX NP group, and TF-PEG-DSPE/DOX NP group. The model mice of each group were treated differently by tail vein injection of drugs, and the corresponding drugs were injected at 4.0 mg/kg daily.

#### 2.4.3. Distribution Spectrum of Drugs in Body Tissues

The mice in each experimental group were randomly divided into two subgroups according to their body weight. The mice in the first subgroup were sacrificed at 0.5 h after the administration. The tumor tissues, heart, brain, liver, and kidney organs were taken, and the distribution of TF-PEG-DSPE/DOX NPs in the mice was recorded.

#### 2.4.4. Survival Analysis

After regularly treating the mice in the second subgroup, the survival time and weight of the mice in the DOX group, PEG-DSPE/DOX NP group, and TF-PEG-DSPE/DOX NP group were recorded to evaluate the antitumor activity of the drug.

## 3. Results and Discussion

### 3.1. Morphological Characteristics of Composite Nanomedicine

The transmission electron microscopy (TEM) image of TF-PEG-DSPE/DOX NPs is shown in Figure 3. It can be seen from the obtained TEM image (Figure 3(a)) that the TF-PEG-DSPE/DOX NPs are spherical, and the agglomeration of the nanoparticles is not obvious, indicating that the physical and chemical properties of the nanoparticles are stable. The size of TF-PEG-DSPE/DOX NPs was determined to be about 100 nm using a particle size analyzer (Figure 3(b)).

RETRACTED

### 3.2. Determination of the BBB Model

The test results of TF-PEG-DSPE/DOX NPs crossing the BBB *in vitro* model are shown in Figure 4. The data shows that the penetration effect of PEG-DSPE/DOX NPs is not significantly different from that of a single DOX drug at 6.0 h (*P* > 0.05), while the penetration effect of TF-PEG-DSPE/DOX NPs is significantly better than that of DOX and PEG-DSPE/DOX NPs (*P* < 0.05). At 12, 18, and 24 h, the penetration rates of PEG-DSPE/DOX NPs and TF-PEG-DSPE/DOX NPs were higher than those of DOX (*P* < 0.05). Among them, the penetration efficiency of TF-PEG-DSPE/DOX NPs at the 24 h node is as high as 7.79 ± 0.37%. Therefore, the TF-PEG-DSPE/DOX NPs prepared in this experiment have great potential in the treatment of glioma.

### 3.3. Inhibitory Effect of Composite Nanodrugs on U87 Cells

The experimentally observed inhibition rate of TF-PEG-DSPE/DOX NPs on U87 glioma cells is shown in Figure 5. The data graph shows that the inhibitory effect of the drug on U87 is in an increasing relationship with the concentration. In addition, compared with DOX and PEG-DSPE/DOX NPs, the inhibitory effect of TF-PEG-DSPE/DOX NPs on U87 cells is significant (*P* < 0.05), and when the drug concentration is 50 *μ*M, the cell inhibition rate is about 88.23 ± 2.55%. It can be seen that TF-PEG-DSPE/DOX NPs have good antitumor effects.

### 3.4. Cumulative Release of Drugs *In Vitro*

The *in vitro* release curves of different drugs under pH = 7.4 are shown in Figure 6. According to the experimental results, within 0.5–3 h, the release of DOX, PEG-DSPE/DOX NPs, and TF-PEG-DSPE/DOX NPs was faster, and their cumulative release rates were 51.40%, 35.55%, and 40.88%, respectively. The release rate of the drug gradually slowed after 3 h. At 9.0 h and 36 h, the cumulative release rate of DOX and PEG-DSPE/DOX NPs reached a peak and stopped. By 48 h, the *in vitro* release rate of TF-PEG-DSPE/DOX NPs reached the maximum. The results show that the experimentally prepared TF-PEG-DSPE/DOX NPs have excellent sustained release properties and can effectively solve the problem of low DOX bioavailability.

### 3.5. Distribution of Drugs in Body Tissues

Through experiments in mice, this work obtained the tissue distribution of different drugs in mice, and the results are shown in Figure 7; the concentration of DOX, PEG-DSPE/DOX NPs, and TF-PEG-DSPE/DOX NPs in kidney tissue is higher, and this phenomenon is related to the renal excretion mechanism of DOX drugs. But compared with DOX (Figure 7(a)), PEG-DSPE/DOX NP group mice (Figure 7(b)) and TF-PEG-DSPE/DOX NP group mice (Figure 7(c)) had lower drug concentration in kidney tissue, which greatly reduces the burden on the kidneys of the body. In addition, the concentration of TF-PEG-DSPE/DOX NPs in the brain tissue is higher than that of DOX and PEG-DSPE/DOX NPs, which indicates that the experimentally synthesized nanoparticles have targeting properties and are more suitable for the treatment of glioma.

RETRACTED

### 3.6. Model Survival

The survival record of the model mice after treatment is shown in Figure 8. It can be seen from the survival curve that in the first 10 days of treatment, death occurred in each experimental group. However, since the 12th day, the number of surviving mice in the DOX group decreased sharply, and as of the 30th day after treatment, only one mouse survived. On the contrary, the survival status of mice in the PEG-DSPE/DOX NP group and TF-PEG-DSPE/DOX NP group was significantly better than that in the DOX group. As of the 30th day after treatment, 7 mice survived in the PEG-DSPE/DOX NP group, and 11 mice survived in the TF-PEG-DSPE/DOX NP group. Therefore, it can be seen that the targeting properties of TF-PEG-DSPE/DOX NPs make it exhibit excellent antitumor effects in animal models of glioma.

## 4. Discussion

The degree of malignancy of glioma is well known. At present, although many medical techniques have been applied to the disease management of glioma, the results of practice are often unsatisfactory. For example, DOX is an antibiotic drug, which often appears in cancer treatment programs. However, after a long period of research, it is found that the existence of BBB restricts the antitumor effect of drugs, which points out the research direction for medical personnel [31].

Considering the difficulties at this stage, this project has synthesized a nanodrug (TF-PEG-DSPE/DOX NPs) combined with multiple biomolecules. In the initial stage of the experiment, the morphology of TF-PEG-DSPE/DOX NPs was characterized, and it was found that the nanoparticles were uniform in size and stable in physical and chemical properties. Secondly, *in vitro* drug release experiments show that the sustained release effect of TF-PEG-DSPE/DOX NPs meets expectations. In addition, TF-PEG-DSPE/DOX NPs performed well in penetrating BBB model experiments. Of course, research on the role of TF-PEG-DSPE/DOX NPs in glioma animal models is also being carried out in subsequent experiments. The results show that TF-PEG-DSPE/DOX NPs can effectively prolong the life cycle of glioma mice. In addition, the retention concentration in the kidney tissue of the body decreases while the concentration in the brain tissue increases, indicating the drug's effects on the kidney tissue; the burden is small.

RETRACTED

In summary, *in vivo* and *in vitro* experiments have confirmed the role of TF-PEG-DSPE/DOX NPs in glioma, which provides data for clinicians to optimize treatment plans.

## 5. Conclusion

The low bioavailability of DOX is the main problem that plagues surgeons. This work has made efforts in this regard. *In vitro* experiments prove that the experimentally synthesized TF-PEG-DSPE/DOX NPs can effectively penetrate BBB and have excellent drug sustained release properties. In addition, *in vivo* animal experiments based on BALB/c nude mice have verified the targeted antitumor effect of TF-PEG-DSPE/DOX NPs in the body. Therefore, TF-PEG-DSPE/DOX NPs nanoparticles are just around the corner in the clinical treatment of glioma.

## Figures and Tables

**Figure 1:** The chemical structural picture of doxorubicin.

**Figure 2:** Related experiments based on doxorubicin-loaded targeting nanoparticles (TF-PEG-DSPE/DOX NPs).

**Figure 3:** Characterization of TF-PEG-DSPE/DOX NPs. (a) Transmission electron microscopy (TEM) image of TF-PEG-DSPE/DOX NPs. (b) Particle size distribution chart of TF-PEG-DSPE/DOX NPs.

**Figure 4:** Effect of nanomedicine crossing the blood-brain barrier *in vitro*.

**Figure 5:** Inhibitory effect of Adriamycin-loaded targeting nanoparticles on U87 glioma cells.

**Figure 6:** The cumulative *in vitro* release of the drug.

**Figure 7:** Tissue distribution of different drugs in mice. (a) DOX. (b) PEG-DSPE/DOX NPs. (c) TF-PEG-DSPE/DOX NPs.

**Figure 8:** Survival records of mice in each group.

## Data Availability

The data underlying the results presented in the study are available within the manuscript.

## References

[1] Zhao W. Y., Zhang C. X., Liu L. (2016). Construction of functional targeting daunorubicin liposomes used for eliminating brain glioma and glioma stem cells. *Journal of Biomedical Nanotechnology*.

[2] Selvapandian A., Manivannan K. (2018). Fusion based glioma brain tumor detection and segmentation using ANFIS classification. *Computer Methods and Programs in Biomedicine*.

[3] Liu Z. H., Tong L., Chen L. (2021). CANet: context aware network for brain glioma segmentation. *IEEE Transactions on Medical Imaging*.

[4] Liu L. Q., Feng L. F., Nan C. R., Zhao Z. M. (2018). CREB3L1 and PTN expressions correlate with prognosis of brain glioma patients. *Bioscience Reports*.

[5] Guo Q. L., Hua W., Wu B. W. (2020). Lateral or medial surgical approaches for thalamic gliomas resection?. *World Neurosurgery*.

[6] Barone F., Alberio N., Iacopino D. G. (2018). Brain mapping as helpful tool in brain glioma surgical treatment toward the perfect surgery. *Brain Sciences*.

RETRACTED

[7] Alimohamadi M., Shirani M., Shariat Moharari R. (2016). Application of awake craniotomy and intraoperative brain mapping for surgical resection of insular gliomas of the dominant hemisphere. *World Neurosurgery*.

[8] Almasian M., Wilk L. S., Bloemen P. R., Van Leeuwen T. G., Ter Laan M., Aalders M. C. G. (2019). Pilot feasibility study of in vivo intraoperative quantitative optical coherence tomography of human brain tissue during glioma resection.. *Journal of Biophotonics*.

[9] Di N. N., Cheng W. N., Jiang X. Y. (2019). Can dynamic contrast-enhanced MRI evaluate VEGF expression in brain glioma? An MRI-guided stereotactic biopsy study. *Journal of Neuroradiology*.

[10] Wang Q., Zhang J. S., Li F. Y., Chen X. L., Xu B. N. (2021). The utility of magnetic resonance spectroscopy in frame-less stereotactic needle biopsy of glioma. *Journal of Clinical Neuroscience*.

[11] Abdelaziz O., Eshra M., Belal A., Elshafei M. (2016). Diagnostic value of magnetic resonance spectroscopy compared with stereotactic biopsy of intra-axial brain lesions. *Part A, Central European neurosurgery*.

[12] Slomski A. (2017). Recombinant influenza vaccine more effective in older adults. *The Journal of the American Medical Association*.

[13] Thome I., Lacle R., Voß A. (2020). Neoplastic cells are the major source of MT-MMPs in IDH1-mutant glioma, thus enhancing tumor-cell intrinsic brain infiltration. *Cancers*.

[14] Massey S. C., Rockne R. C., Hawkins-Daarud A. (2018). Simulating PDGF-driven glioma growth and invasion in an anatomically accurate brain domain. *Bulletin of Mathematical Biology*.

[15] Wright A. J., Fellows G., Byrnes T. J. (2009). Pattern recognition of MRSI data shows regions of glioma growth that agree with DTI markers of brain tumor infiltration. *Magnetic Resonance in Medicine*.

[16] Robinson M. H., Vasquez J., Kaushal A. (2020). Subtype and grade-dependent spatial heterogeneity of T-cell infiltration in pediatric glioma. *Journal for Immuno Therapy of Cancer*.

[17] Taffelli A., Amelio D., Fellin F. (2018). 48. Dosimetric predictors of radiation induced alopecia in brain tumours proton therapy. *European Journal of Medical Physics*.

[18] Harahap Y., Ardiningsih P., Winarti A., Purwanto D. (2020). Analysis of the doxorubicin and doxorubicinol in the plasma of breast cancer patients for monitoring the toxicity of doxorubicin. *Drug Design, Development and Therapy*.

[19] Lin Y. R., Wu C. E., Huang M. F. (2017). Development of doxorubicin quantification by reductive amination. *Current Analytical Chemistry*.

RETRACTED

[20] Wen S. H., Su S. C., Liou B. H., Lin C. H., Lee K. R. (2018). Sulbactam-enhanced cytotoxicity of doxorubicin in breast cancer cells. *Cancer Cell International*.

[21] Eide S., Feng Z. P. (2020). Doxorubicin chemotherapy-induced “chemo-brain”: meta-analysis. *European Journal of Pharmacology*.

[22] Chen X. X., Yuan M. Q., Zhang Q. Y., Yang Y. T., Gao H. L., He Q. (2016). Synergistic combination of doxorubicin and paclitaxel delivered by blood brain barrier and glioma cells dual targeting liposomes for chemotherapy of brain glioma. *Current Pharmaceutical Biotechnology*.

[23] Li X. H., Wang X. J., Xie J. W., Liang B., Wu J. H. (2019). Suppression of angiotensin-(1–7) on the disruption of blood-brain barrier in rat of brain glioma. *Pathology & Oncology Research*.

[24] Firkins J., Ambady P., Frank J. A., Neuwelt E. A. (2018). Safety of intra-arterial chemotherapy with osmotic opening of the blood brain barrier. *Journal of Clinical Oncology*.

[25] Nair L. V., Nair R. V., Shenoy S. J., Thekkuveettil A., Jayasree R. S. (2017). Blood brain barrier permeable gold nanocluster for targeted brain imaging and therapy: an in vitro and in vivo study. *Journal of Materials Chemistry B*.

[26] Stocki P., Szary J., Rasmussen C. L. M. (2021). Blood-brain barrier transport using a high affinity, brain-selective VNAR antibody targeting transferrin receptor 1. *The FASEB Journal*.

[27] Moos T., Morgan E. H. (2000). Transferrin and transferrin receptor function in brain barrier systems. *Cellular and Molecular Neurobiology*.

[28] Johnsen K. B., Burkhart A., Melander F. (2017). Targeting transferrin receptors at the blood-brain barrier improves the uptake of immunoliposomes and subsequent cargo transport into the brain parenchyma. *Scientific Reports*.

[29] Wang Y. Z., Fan W., Dai X. (2014). Enhanced tumor delivery of gemcitabine via PEG-DSPE/TPGS mixed micelles. *Molecular Pharmaceutics*.

[30] Wang R., Xiao R., Zeng Z., Xu L., Wang J. (2012). Application of poly(ethylene glycol)-distearoylphosphatidylethanolamine PEG-DSPE block copolymers and their derivatives as nanomaterials in drug delivery. *International Journal of Nanomedicine*.

[31] Kundu M., Das S., Dhara D., Mandal M. (2019). Prospect of natural products in glioma: a novel avenue in glioma management. *Phytotherapy Research*.

